# Circadian Period 2 (Per2) downregulate inhibitor of differentiation 3 (Id3) expression via PTEN/AKT/Smad5 axis to inhibits glioma cell proliferation

**DOI:** 10.1080/21655979.2022.2074107

**Published:** 2022-05-21

**Authors:** Yifan Zhang, Xvlei Hu, Hailiang Li, Jian Yao, Ping Yang, Yuanxiang Lan, Hechun Xia

**Affiliations:** a School of Clinical Medicine, Ningxia Medical University, Yinchuan, China; b Ningxia Human Stem Cell Institute, General Hospital of Ningxia Medical University, Yinchuan, China; c Department of Neurosurgery, Ningxia Human Stem Cell Institute, General Hospital of Ningxia Medical University, Yinchuan, China

## Abstract

In this study, we employed multiple laboratory techniques to acknowledge the biological activities and processes of Per2 and Id3 in glioma. We analyzed TCGA and CGGA databases for seeking association among Per2, Id3, and clinical features in glioma. Immunohistochemistry and Western blot were used to detect protein expression levels. CCK-8 assay, colony formation assay, Transwell assay, the wound healing assay, flow cytometric, and Xenograft nude mice were used to acknowledge the impact of Per2 and Id3 on biological behavior of glioma. The results showed that the Per2 mRNA expression was negatively correlated with the WHO grade, while the Id3 mRNA expression was positively correlated with the WHO grade in patients with glioma in TCGA and CGGA databases. Per2 and Id3 maintained separate prognostic abilities and had a negative connection in human glioma. In the clinical sample study, Per2 and Id3 were validated at the protein level with the same results compared to the mRNA expression level in TCGA and CGGA. By using a wide range of functional examples, overexpression of Per2 restrains malignant biological behaviors in glioma cells by many ways, while Id3 promotes malignant biological behaviors in glioma cells. Furthermore, overexpression of Per2 can inhibit Id3 expression via regulating PTEN/AKT/Smad5 signaling pathway and thereby abolish malignant biological behaviors that are caused by Id3 overexpression. These results suggested that Per2 inhibits glioma cell proliferation through regulating PTEN/AKT/Smad5/Id3 signaling pathway, which may be a viable therapeutic target for glioma.

## Highlight

- Per2 was negatively correlated with the WHO grade and had a better prognosis based on databases and clinical samples.
- Id3 was positively correlated with the WHO grade and had a poor prognosis based on databases and clinical samples.
- Per2 counteracts malignant growth by affecting PTEN/AKT/Smad5 signaling pathway to downregulate Id3 expression.

## Introduction

Glioma is the most common central nervous system tumors emerging from glial or their precursors, accounting for approximately 25.5% of all primary brain and other CNS tumors and 80.8% of malignant tumors, glioblastoma (GBM), the most malignant glioma, accounts for 57.3% of gliomas. Furthermore, the five-year survival rate for malignant glioma is approximately 51.4%, while that for GBM is a mere 6.8% [1]. In the past, the most effective conventional treatments of glioma are surgical resection, radiation, and chemotherapy. Varied over time, with the significant improvements resulting from chemotherapy and surgical advances, the two-year survival rate for GBM has been improved approximately 2.7% for the past 16 years, primarily due to treatment with temozolomide (TMZ). However, the therapeutic effect is still unsatisfactory [2]. In addition, due to the infiltrative nature of malignant glioma and on the verge of eloquent brain regions, surgical excision with a margin of healthy tissue is very difficult to achieve, and even with the best standards of treatment, including chemotherapy and radiation therapy, tumor recurrence is often inevitable [3].As a result, new insights into glioma are being discovered. A novel treatment immunotherapy, which exhibits potent effects in lung cancer and melanoma. However, it only works for specific groups and has an inadequate clinical study in glioma patients [4]. Along with technical advancements, progress in the knowledge of gliomas at the molecular level has led to the discovery of significant genetic mutations in gliomas, which contribute to the discovery of novel treatments for glioma. To search targeted drugs and better targeted therapies for patients, panel, whole-exome, and whole-genome sequencing are becoming increasingly popular methods of discovery [5]. But in patients with brain tumors, genomics has not yet delivered on its promise of discovering novel therapeutic targets. As a result, we must continue to seek new drug targets and understand the biology of drug targets to increase the therapeutic efficacy of glioma chemotherapy [6].

The circadian clock, metabolism, metabolic syndrome, and associated illnesses have all been implicated in previous investigations as being linked at the molecular level [7]. Breaking the circadian clock has a large effect on cells division and cancer origin, which affects cancer in a tissue-specific way [8]. Circadian clock disturbances are closely associated with multiple tumor types, such as melanoma, pancreatic cancer, colorectal cancer, lymphoma, prostate cancer, non-small-cell lung cancer, breast cancer, glioma, and gastric cancer [9]. The PER proteins represent the first regulatory limb of the circadian clock and function as negative regulators of CLOCK–BMAL1 [10]. Period 2 (Per2) belongs to the Period family, which also includes Period 1 (Per1), Period2 (Per2), and Period3 (Per3), and the brain and external nervous systems are the primary expression sites [11]. Multiple studies have found that Per2 appears to primarily mediate antitumorigenic programs, especially in gliomas [12]. Our previous studies further reinforced that in glioma and glioma stem cells (GSCs), Per2 plays a vital role in the biological mechanism of malignant progression [13,14]. Furthermore, the PI3K/AKT/mTOR pathway is affected by Per2 in oral squamous cell carcinoma, demonstrating that Per2 is a tumor suppressor in multiple mechanistic investigations [15]. Per2 also can affect PTEN/PI3K/AKT signaling pathway in osteoarthritis [16]. They suggested that Per2 may target PTEN/AKT pathway in various diseases.

Tumorigenesis and development are related to a multitude of variables, with inhibitor of differentiation (ID) proteins, in particular, being shown to have a significant role in the advancement of various neoplasms. The Id family of transcription factors (Id1, Id2, Id3, and Id4) is an element of the basic helix-loop-helix (bHLH) family of transcription factors that regulate stem cell maintenance and fate commitment in a variety of cell types [17]. Id proteins play a role in several stages of carcinogenesis by espousing numerous essential characteristics of tumor growth (deregulated proliferation, invasiveness, angiogenesis, and metastasis) and activating oncogenic pathways. Id proteins transmit embryonic stem cell phenotypes to cancer cells leading to aberrant activation [18]. Increasing evidence suggests that dysregulation of Id proteins, particularly Id1, Id2, and Id3, is related to advanced tumor grade and a dismal prognosis in a wide range of human cancers [19]. According to recent research, Id3 is correlated with tumor grades in human astrocytes [20] and is downstream of the EGFR/AKT/Smad5 pathway [21]. But the role of Id3 research is insufficient and needs further to clarify its effects on proliferation and invasion in glioma.

Here, we aim to explore whether overexpression of Per2, a tumor suppressor gene, may inhibit the malignant phenotype of glioma based on regulating PTEN/AKT/Smad5/Id3 signaling pathway and would help to identify a novel target for clinical precision medicine.

## Material and methods

### Clinical samples

Fifty-nine paraffin-embedded samples were obtained from patients who were diagnosed with glioma and underwent tumor excision between February 2014 and November 2016. The samples utilized in this investigation were collected at the General Hospital of Ningxia Medical University. None of the patients had received any preoperative chemotherapy or radiation in the preceding year. The time between surgery and death, or the end of the research period, was used to calculate overall survival (OS). Informed consent forms were signed by all patients. The Ethical Committee of Ningxia Medical University approved this investigation.

### Bioinformatics analysis

Data from glioma patients, including clinical characteristics and mRNA levels of Per2 and Id3, were collected from The Cancer Genome Atlas (TCGA) database and the Chinese Glioma Genome Atlas (CGGA). TCGA (https://portal.gdc.cancer.gov/) and CGGA (http://www.cgga.org.cn/) are open to the public, and no ethics approval was required to access these data.

### Cell culture and pretreatment

Human glioma U87 and U251 cells were obtained from the Cellcook Biology Company (Guangzhou, China) and were last authenticated using short tandem repeat (STR) profiling in 2021. In all cases, cell lines were grown in DMEM (Gibco, CA, USA) supplemented with 10% FBS (Gibco-BRL) and 1% antibiotics (0.1 um Triple Sterile Filtered, Penicillin 10,000 units/ml, Streptomycin 10,000 ug/ml, SEVEN Beijing, China). Bisperoxovanadium(bpV) (SML0884, Sigma-Aldrich) 2 μM, a potent and selective inhibitor of PTEN, were used to pretreat Per2 OE cells for 24 h. AKT activator SC79 (SML0749, Sigma-Aldrich) 10 μM were used to pretreat Per2 OE cells for 12 h.

### Lentivirus transduction

Overexpressed Per2 and Id3 in lentivirus form were obtained from Gene Chem Co, Ltd, (Shanghai, China). The U87 and U251 cells were infected with Per2-GFP lentiviral particles and Id3-mCherry lentiviral particles. U87 and U251 cells were fixed with 4% paraformaldehyde, and PBS were used to wash for three times. A solution of 4ʹ,6- diamidino-2-phenylindole (DAPI) (ZLI-9557, ZSGB-BIO, China) was used to stain nuclei. they were validated by Fluorescence microscope.

### Immunohistochemistry (IHC)

IHC was performed by two independent pathologists using a modified Histo-score (H-score). The 59 glioma tissue slides were handled with Per2 antibodies (1:200, Abcam, ab200388) and Id3 antibodies (1:200, BIOSS, bs-6229R), which were purchased from Abcam (USA) and BIOSS (Beijing, China). The immunoreactive score (IRS) calculation was performed by multiplying the staining intensities by the percentage scores of positive cells, with scores varying from 0 to 12. The intensity of the staining was graded as follows: 0 (no staining), 1 (weak staining), 2 (moderate staining), and 3 (strong staining), and the percentages of positive cells were scored as follows: 0 (0%), 1 (1%–25%), 2 (26%–50%), 3 (51%–75%), and 4 (76%–100%) [22].

### Western blotting

After plating U87 and U251 cells in six-well plates, RIPA buffer (KeyGen, Jiangsu, China) was added to lyse the cells on a 4°C shaker for approximately 10 minutes, and cells were subsequently scraped off the six-well plates into EP tubes, which were placed on a 4°C shaker for approximately 30 minutes. Next, the lysates were subjected to 15-minute centrifugation at 12,000 rpm to remove residue. Protein concentrations were determined using the BCA Protein Assay Kit (KeyGen, Jiangsu, China). SDS-PAGE was used to separate the protein extracts, which were then transferred onto polyvinylidene difluoride (PVDF) membranes, followed by incubation with the following primary antibodies overnight on 4°C shakers: Per2 (Abcam, ab179813), Id3 (Abbkine, ABP58864), PTEN (BIOSS, bsm-52369R), AKT (Proteintech, 60203-2-Ig), p-AKT (T308) (Proteintech, 29163-1-AP), p-AKT (S473) (Proteintech, 80455-1-RR), Smad5 (BIOSS, bs-13890R), p-Smad5 (BIOSS, bs-19918R), GAPDH (BIOSS, bsm-33033M) and β-tubulin (Zen Bioscience Chengdu, China, 200608). The membranes were incubated with secondary antibodies the next day (goat anti-mouse 926–32210, goat anti-rabbit 926–32211, LI-COR, USA) for 2 hours at ambient temperature before detection.

### Cell proliferation and colony formation assay

The Cell Counting Kit-8 was used to determine cell proliferation rate (CCK-8, Trans, Beijing, China). A cell density of 6000 cells per well was used to plate the transfected cells into 96-well plates, where they were cultured for 48 hours. The absorbance was subsequently measured at 450 nm for 12 h, 24 h, 36 h, and 48 h, and the OD values were recorded. For the colony formation experiment, a total of 1*103 cells were dispersed onto six-well plates for incubating 14 days. 0.5% crystal violet was used to stain cells for 10 minutes after 4% paraformaldehyde-fixed for 30 minutes. It was considered a clone when the number of cells was greater than 50 under the light microscope.

### Cell migration and invasion assay

Experiments were conducted using Corning 24-well Transwell chambers (Corning, Bedford, MA, USA) with or without Matrigel (Corning). For this experiment, 2*104 cells were plated in 200 ul serum-free DMEM into the upper chambers, and 500 uL 20% FBS media was placed into the bottom chambers. A 24-hour incubation period was followed by a 30-minute fixation step in 4% paraformaldehyde and 10-minute crystal violet staining step in 0.1% crystal violet. Cells were counted using ImageJ software (Rawak Software Inc. Stuttgart, Germany).

### Wound healing assay

The wound healing assay was utilized to assess cell mobility. Briefly, six-well plates were seeded with glioma cells. Using 200 ul pipette tips, several scratches were made in the cell monolayers when cell density was approximately 90%. Next, the previous culture solution was treated for one hour with mitomycin (1 ug/ml) to suppress cell growth. Afterward, the previous culture solution was removed and washed three times in PBS before being replaced with 2 ml of serum-free medium. An inverted microscope (Olympus) was used to obtain images at 0 h and 48 h.

### Flow cytometry analysis

To determine the cell cycle distribution, U87 and U251 cells were cultured for 48 h to 70%-80% confluence, at which point trypsin was added to detach cells, and they were centrifuged twice at 1000 rpm for 5 min, which was repeated by adding PBS to the first pellet. Cells were collected in 1.5 ml EP tubes, according to the protocol of the Cell Cycle Staining Kit (MultiSciences, Hangzhou, China), the PI staining solution with RNase A was applied and incubated for 30 min in the dark at 37°C. Stained samples were examined using a BD FACSCalibur™ Flow Cytometer (BD Biosciences), and data were interpreted using ModFit LT software for Windows (Version 5.0.9).

### Xenografts in nude mice

Male BALB/c nude mice (4–5 weeks old) were randomly assigned to four groups with six mice each. Approximately 1 × 105 transfected U87 cells (U87-control-luciferase, U87-Per2 OE-luciferase, U87-Id3 OE-luciferase, or U87-Id3 OE+Per2 OE-luciferase) were intracranially injected into in the right prefrontal cortex of mice. D-fluorescein 150 g/g was intraperitoneally administered to the animals following anesthesia for xenogeny bioluminescence imaging. Eventually, the mice were euthanized due to growing tumor burden-induced neurological impairment. In accordance with the Care and Use of Laboratory Animals, Ningxia Medical University’s Ethical Committee approved all animal research at the university.

### Statistical analysis

GraphPad 8 and RStudio 4.0.3 were used for statistical analysis. The R statistical tool was used to construct box plots using TCGA and CGGA data. Two groups were compared using Student’s t-test. One-way ANOVA was used to compare more than two groups. Kaplan–Meier survival analysis was used to compare the survival rates of patients in the high- and low-expression groups based on the 50% cutoff point. Univariate analysis and multivariate analysis were utilized to identify independent variables impacting patients’ prognosis. Pearson’s test was employed to assess the connection between genes. Discontinuous variables are shown in terms of the number of instances and percentage (%) or composition ratio, and the chi-square test was employed for comparisons between groups. Statistical significance was defined as p < 0.05.

## Results

In this study, we analyzed the clinical significance and relevance of Per2 and Id3 in patients with glioma using bioinformatics combined with immunohistochemistry of clinical samples. Next, CCK8, colony formation, Transwell, wound healing assay, flow cytometry and xenografts in mice were used to acknowledge the effect of Per2 and Id3 in glioma. In addition, we clarified the mechanism of Per2 affecting Id3 expression by western blot.

### Per2 and Id3 expression levels in human glioma predict patient prognosis

To assess the relationship between two genes and the WHO grade, chi-square test of the original data from TCGA and CGGA revealed that abnormally high mRNA expression of Per2 was negatively correlated with the WHO grade, while high mRNA expression of Id3 was positively correlated with the WHO grade in patients with glioma (Figure 1a, FigureS1a). Then, we performed survival analysis using these two datasets, revealing that patients with high mRNA expression of Per2 exhibited longer survival, whereas patients with high mRNA expression of Id3 displayed poorer survival (Figure 1b, Figure S1b). When the TCGA and CGGA datasets were combined, it was discovered that Per2 and Id3 still maintained separate prognostic abilities (Figure 1c, d, Figure S1c, d). The databases were next used to examine the correlations between mRNA levels of Per2 and Id3, which revealed that they were inversely correlated in human glioma (Figure 1e, Figure S1e).

**Figure 1.** Per2 and Id3 mRNA expression in glioma based on CGGA. (a) Correlation analysis of Per2 and Id3 with glioma grade. (b) Kaplan–Meier survival analysis with respect to Per2 and Id3. (c) Univariate and multivariate Cox regression of Per2. (d) Univariate and multivariate Cox regression of Id3. (e) Relationship between Per2 and Id3 of mRNA expression level.

### Per2 and Id3 expression levels in gliomas tissue from clinical samples

The protein levels of Per2 and Id3 in 59 glioma specimens were assessed using IHC. The immunoreactive scores of glioma samples were divided into high expression and low expression groups using the median score as the cutoff. As such, an IRS of Per2 > 4 defined high expression, while ≤4 defined low expression, and an IRS of Id3 > 8 defined high expression, while ≤8 defined low expression. The percentage of high and low expression of each gene in WHO grade was compared, and we discovered that Per2 was negatively correlated with WHO grade (F = 10.67, df = 1), whereas Id3 was positively correlated with WHO grade (F = 11.68, df = 1) (Figure 2c). Next, we examined overall survival based on protein expression levels and found that high Per2 expression was associated with longer survival than low Per2 expression, whereas high Id3 expression was associated with shorter survival than low Id3 expression (Figure 2d). The representative IHC images of Per2 and Id3 in different pathological grades of glioma tissue were displayed in Figure 2a, b. Further investigation of the association between the two proteins revealed that they were negatively correlated in glioma tissue, consistent with database analysis (Figure 2e). Based on these findings, we hypothesized that Per2 is involved in Id3 expression in gliomas, which we explored in subsequent experiments.

**Figure 2.** Per2 and Id3 protein expression in clinical samples. (a) Images of Per2 IHC staining in various grades of glioma tissue (scale bar, 100 μm). (b) Images of Id3 IHC staining in various grades of glioma tissue (scale bar, 100 μm). (c) Correlation analysis of Per2 and Id3 with glioma grade. (d) Kaplan–Meier survival analysis with respect to Per2 and Id3. (e) Relationship between Per2 and Id3 of IRS levels.

### Overexpression of Per2 restrains proliferation, migration, invasion, and cell cycle progression in vitro

Per2 was stably overexpressed (Per2 OE) in U87 and U251 cells using lentiviral vector transfection to assess the functional consequences of increasing levels of Per2 in glioma, while empty lentiviral vector-transfected cells served as controls. The infection efficiency of Per2 lentiviral vector was validated by fluorescence microscope (Figure S2a, b). The protein levels of Per2 were validated using western blotting (Figure 3a. Figure S3a). The CCK8 assay and the colony formation assay showed that Per2 OE inhibited the proliferation of glioma cells (Figure 3b, c. Figure S3b, c). Then, we examined migration and invasion using Transwell and Matrigel assays, and Per2 OE impaired both migration and invasion abilities (Figure 3d. Figure S3d). The wound healing assay was used to determine the motility of glioma cells, and Per2 OE hindered migration to some extent (Figure 3e. Figure S3e). In addition, flow cytometry was used to analyze the influence of Per2 OE on U87 and U251 cells. The results illustrated that the percentage of S-phase cells had declined, and cells were arrested in the G0/G1 cycle in response to Per2 OE, while the G2/M phase was not markedly changed (Figure 3f. Figure S3f). In summary, Per2 OE restrains proliferation, migration, invasion, and cell cycle progression, indicating the tumor suppressor role of Per2 in glioma cells.

**Figure 3.** Effect of Per2 overexpression and Id3 overexpression in U87 cells. (a) Western blot examination of Per2 protein expression in U87 cells transfected with lentiviral vector. (b) The CCK-8 assay revealed the impact of Per2 overexpression on proliferation. (c) The cell proliferation was assessed by colony formation. (d) Migration and invasion measured by Transwell assay. (e) Migration was assessed by the wound healing assay (scale bar, 200 μm). (f) Cell cycle progression was analyzed by flow cytometry. (g) Western blot examination of Id3 protein expression in U87 cells transfected with lentiviral vector. (h) The CCK-8 assay revealed the impact of Id3 overexpression on proliferation in U87 cells. (i) The cell proliferation was assessed by colony formation. (j) Migration and invasion measured by Transwell. (k) Migration was assessed by the wound healing assay (scale bar, 200 μm). (l) Cell cycle progression was analyzed by flow cytometry. For each assay, three separate tests were conducted. *P < 0.05, **P < 0.01 vs. control group.

### Id3 promotes proliferation, migration, invasion and cell cycle progression

Next, we investigated the impact of Id3ʹs overexpression on glioma cells. Similarly, we employed lentiviral vector transfection of Id3 overexpression (Id3 OE). The infection efficiency of Id3 lentiviral vector was validated by fluorescence microscope (Figure S2c, d). The protein levels of Id3 was validated using western blotting (Figure 3g. Figure S3g). In response to Id3 OE, the CCK-8 assay and colony formation revealed dramatically boosted cell proliferation (Figure 3h, i. Figure S3h, i). Previously mentioned techniques were used to assess migration and invasion, and Id3 OE upregulated the invading cell populations compared to controls (Figure 3j. Figure S3j). Similarly, wound-healing experiments confirmed that Id3 OE increases motility (Figure 3k. Figure S3k). Using flow cytometry to examine cell cycle progression, the percentage of S-phase was increased in U87 and U251 cells, G0/G1 phase was decreased, and G2/M phase exhibited slight oscillations (Figure 3l. Figure S3l).

### Per2 suppresses Id3 expression in U87 and U251 cells

To validate that Id3 is downstream of Per2, we examined the impact of Per2 OE on Id3. Western blot analysis demonstrated that Per2 OE reduced Id3 expression in U87 and U251 cells, whereas Id3 OE did not affect expression levels of the Per2 protein (Figure 4a, Figure S4a). Collectively, these data suggest that Per2 suppresses Id3 expression in U87 and U251 cells.

**Figure 4.** Per2 overexpression affects the cell phenotype by regulating Id3 expression in U87 cells. (a) Per2 overexpression decreased Id3 expression, but Id3 overexpression did not affect expression levels of Per2 protein. (b) The CCK-8 assay was used to assess proliferation. (c) The cell proliferation was assessed by colony formation. (d) Migration and invasion measured by Transwell assay. (e) The wound healing assay. (f) The cell cycle progression of variation. *P < 0.05, **P < 0.01, ***P < 0.001 vs. control group. ^#^P < 0.05, ^##^P < 0.01, ^###^P < 0.001 vs. Id3 OE.

### Per2 suppresses proliferation, migration, invasion and cell cycle progression by regulating Id3 expression in U87 and U251 cells

To illustrate that Per2 controls the development of glioma by suppressing Id3, we first overexpressed Id3 in U87 and U251 cells and then transfected a lentiviral vector overexpressing Per2 in Id3 OE cells (Id3 OE+Per2 OE) to confirm that Per2 can reverse the Id3-mediated malignant biological behavior of glioma. The co-infection efficiency of lentiviral vector was validated by fluorescence microscope (Figure S2e, f). We discovered that Id3 OE caused glioma cells to proliferate faster than controls in CCK-8 assays and colony formation, while proliferation was inhibited when the transfected Per2 OE vector was present (Figure 4b, c, Figure S4b, c). The same phenomenon was observed in migration and invasion using Transwell assays and wound healing assay (Figure 4d, e, Figure S4d, e). Using flow cytometry to assess cell cycle progression, Per2 was shown to affect the percentage of S-phase of Id3 OE cells by shifting them to the G0/G1 phase, while the G2/M phase exhibited no significant variation (figure 4f, Figure S4f).

### Per2 overexpression reduces tumor formation and improves survival in nude mouse xenograft model

To determine whether the influence of Per2 overexpression can be similarly verified in vivo, we created U87-Per2 OE cells, U87-Id3 OE cells, U87-Id3 OE+Per2 OE cells, and U87-empty lentiviral vector cells as controls, and tumor cells were intracranially transplanted into nude mice to assess tumorigenesis. After 4 weeks, IVIS (in vivo imaging system) analysis showed that U87-Per2 OE tumor size was less than control, the U87-Id3 OE group was obviously larger than control, while the U87-Id3 OE+Per2 OE group was visibly restrained compared to the U87-Id3 OE group, suggesting that Per2 OE slows tumor growth (Figure 5a, b). According to survival comparison, the Per2 OE group exhibited extended survival compared to the control group, while the Id3 OE group died earlier. Similarly, the U87-Id3 OE+Per2 OE group’s survival was prolonged compared to the Id3 OE group (Figure 5c). Taken together, these data show that Per2 mitigates glioma development by downregulating Id3.

**Figure 5.** Effect of Per2 overexpression in vivo. (a) Xenograft (4 weeks) measured by IVIS. (b) Quantification of photo flux separately. (c) Overall survival of mice was calculated using Kaplan–Meier survival curves. *P < 0.05, **P < 0.01 vs. control group. **^#^**P < 0.05 vs. Id3 OE.

### Per2 inhibit Id3 expression via regulating PTEN/AKT/Smad5 signaling pathway

As Per2 can promote PTEN expression [16], and PTEN slack AKT phosphorylation [23]. What’s more, Id3 was the downstream of AKT/Smad5 [21]. All in all, we have reason to believe that Per2 affecting Id3 by PTEN/AKT/Smad5 axion. To clarify above mechanism in glioma, we measured protein levels of PTEN, AKT, p-AKT (T308), p-AKT (S473), Smad5, and p-Smad5 by using Western blot in glioma cells. Per2 OE activated PTEN expression. Meanwhile overexpression of PTEN inhibited p-AKT (T308), p-AKT (S473), and p-Smad5. To further acknowledge that Per2 directly motivates PTEN expression, we used PTEN inhibitor Bisperoxovanadium (bpV) and AKT activator (SC79) separately. PTEN was downregulated when Per2 OE was pretreated with bpV, and p-AKT (T308), p-AKT (S473), and p-Smad5 were upregulated. PTEN had no variation when Per2 OE pretreated with SC79, while p-AKT (T308), p-AKT (S473), and p-Smad5 were upregulated (Figure 6).

**Figure 6.** Per2 inhibit Id3 expression via regulating PTEN/AKT/Smad5 signaling pathway. The protein levels of PTEN, AKT, p-AKT(T308), p-AKT(S473), Smad5, p-Smad5, GAPDH were analyzed by Western blot in U87 and U251 cells.

## Discussion

An increasing number of researchers are investigating the function of the circadian clock in pathologies such as inflammation, cancer, and dementia. Only a few studies have focused on the Period gene and glioma, particularly in clinical sample merging databases. Previously, we utilized MRS and DWI to measure cell proliferation to gauge the grade of glioma in a laboratory setting, which had a positive impact on appraisal [24]. In this study, Per2 and Id3 were expressed in glioma tissues and were shown to be associated with patient outcomes in glioma patients. We investigated the downstream processes of Per2 and discovered that Per2, a tumor suppressor gene, inhibited glioma cell proliferation by downregulating Id3 expression in glioma.

Initially, we investigated the TCGA and CGGA databases and discovered that Per2 and Id3 are associated with the WHO glioma grade, 5-year survival rate, and prognostic risk, and the two genes appear to be negatively correlated with each other. In TCGA, we discovered that the HR values of the two proteins are consistent with the trend in CGGA but had no significant difference. In comparison, both of them had significant difference in CGGA. A recent study reported a close association between higher PER expression and better overall survival for IDH-mutated or wild-type samples in TCGA, and PER expression was shown to be an independent prognostic factor in glioma according to a Cox proportional hazards analysis with the glioma microenvironment influencing PER expression. But the level of PER expression obtained from the average of PER1/2/3 expression reflected overall PER expression in the research rather than the level of subgenes [25]. Previous research indicated that Per2 is highly expressed in low-grade glioma and exhibits low expression in high-grade glioma in clinical samples [26]. Our finding of the clinical sample is compatible with previous research, and the survival analysis in the clinical sample is also consistent with database survival analysis in TCGA and CGGA. Previous, we found that the cell proliferation, migration, and invasion of Nasopharyngeal carcinoma (NPC) are all inhibited when Period 2 is overexpressed, as we observed in vitro and in vivo, and overexpression of PER2 has been shown to boost the chemotherapeutic effectiveness of a new nanosystem that includes 10-hydroxycamptothecin (HCPT) [27]. Similarly, in non-small cell lung cancer, Per2 overexpression inhibits proliferation, migration, invasion, and cell cycle progression [28]. Another study discovered that Per2 may influence glycolytic gene expression to affect lung cancer growth [29]. Wang *et al* [30] confirmed that Per2 suppresses ovarian cancer growth and metastasis in vivo and that Per2 exhibits similar antitumor effects in other cell types [31]. The same results were achieved in our study with glioma cells in vitro and in vivo models, but we did not examine the particular mechanism by which Per2 reduces malignancies by modifying metabolism.

There are few studies on the biological function of Id3, particularly in glioma. Previous research has shown that tumor xenograft neurogenesis, angiogenesis, and vascularization are dependent on Id1 and Id3, and Id3 is especially crucial for tumor angiogenesis [32]. Huang *et al* demonstrated that Id3 is a critical factor for stemness maintenance in Intrahepatic Cholangiocarcinoma, and high expression of Id3 enhances chemoresistance [33]. Vandeputte DA discovered Id3 expression to be highly correlated with WHO glioma grade in prior work but did not investigate whether it could be an independent prognostic factor [20]. Based on the TCGA and CGGA databases, our research revealed that it is negatively correlated with prognosis and survival, and clinical samples confirmed this finding. In the carcinogenesis and progression of esophageal squamous cell carcinoma, overexpression of Id3 promotes tumor expansion, migration, and invasion, while knockdown of Id3 seems to attenuate these effects, indicating that Id3 is a cancer promoter [34]. As in this study, Id3 owns the same biological function in glioma.

In the study of the influence on the mechanism of Per2, it acts as a vital role in intricate networks and has a significant effect on the PTEN/AKT pathway in a variety of cells. Phosphatase and tension homolog (PTEN) can dephosphorylate phosphatidylinositol 3,4,5-trisphosphate (PIP3), thereby slack AKT phosphorylation [23]. Akt activation is a significant predictor of global histone acetylation levels in glioma cells via Akt-dependent metabolic reprogramming to increase acetyl-CoA synthesis, and histone acetylation level is a valuable biomarker for predicting tumor recurrence [35]. In the previously cited literature [15], Per2 was shown to be involved in the progression of oral squamous cell carcinoma through the PI3K/AKT/mTOR pathway. Similarly, Per2 has the same effect on PI3K/AKT downstream signaling in ovarian cancer [36]. PI3K/AKT is the most common tumor pathway in gliomas and is strongly linked to tumor growth and differentiation; The subunit p85 of PI3K phosphorylates phosphatidylinositol 3,4-bisphosphate (PIP2) which activates catalytic subunit p110, resulting in phosphatidylinositol 3,4,5-trisphosphate (PIP3); when PIP3 phosphorylates Thr308 and the Ser473 residues of the phosphoinositide-dependent kinase (PDK) 1 and Akt, the downstream molecule mTOR is phosphorylated, which causes protein synthesis to be initiated [37]. Sun *et al* [38] found that Id3 was downstream of the AKT pathway, and overexpression of Id3 induced invasion and upregulated MMP2 expression in breast cancer. Meanwhile, Id3 was identified as downstream of the AKT pathway in glioma [21,39]. Based on these findings, we conjecture that Per2 regulates glioma through downstream Id3, and in this study, protein levels of Id3 were reduced when Per2 was overexpressed, while Id3 overexpression did not change the levels of Per2 protein. When Per2 overexpression was induced in glioma cells with Id3 overexpression, Per2 alleviated the increased malignancy of glioma caused by Id3, as shown by multiple experiments. Finally, we studied the connection between Per2 and Id3, and found that Per2 regulate Id3 via PTEN/AKT/Smad5 signaling pathway. However, the limitation is that the driving force of Id3 promoting tumorigenesis in our work requires more investigation.

## Conclusion

In summary, we show that Per2, which had a negative correlation with WHO grade in glioma samples, had a valuable prognosis and better survival from the CGGA and TCGA databases, while Id3, which had a positive correlation with WHO grade in glioma samples, had a poor prognosis and worse survival from the datasets. Per2 inhibits proliferation, migration, invasion, and cell cycle, while Id3 has the opposite effect. Furthermore, we may deduce from the mechanism that Per2 counteracts malignant growth by affecting PTEN/AKT/Smad5 signaling pathway to downregulate Id3 expression. Overall, our findings suggest that Per2 may be a viable therapeutic target for glioma.

## Supplementary Material

Supplemental Material

## Data Availability

The raw data supporting the conclusions of this article will be made available by the authors, without undue reservation.
